The article "The Mechanism of Traditional Chinese Medicine Based on Semi-Targeted Metabolomics to Improve IVF Outcomes in Senile Patients" was published in 2021. Journal: Evid Based Complement Alternat Med.

# The Mechanism of Traditional Chinese Medicine Based on Semi-Targeted Metabolomics to Improve IVF Outcomes in Senile Patients

**DOI:** 10.1155/2021/6696305

**Published:** 2021-11-10

**Authors:** Ying-Jie Ma, Li-Hua Yuan, Ji-Mei Xiao, Hua-Ying Jiang, Yuan-Hong Sa, Hong-Qi Sun, Jing-Yan Song, Zhen-Gao Sun

**Affiliations:** ^1^Shandong University of Traditional Chinese Medicine, Jinan 250014, China; ^2^Reproductive and Genetic Center of Integrated Traditional and Western Medicine, The Affiliated Hospital of Shandong University of Traditional Chinese Medicine, Jinan 250011, China; ^3^Shanghai University of Traditional Chinese Medicine, Shanghai 201203, China; ^4^Heze Hospital of Traditional Chinese Medicine, Heze 274000, China; ^5^Laizhou Maternal and Child Health Hospital of Shandong, Yantai 261400, China; ^6^Qingyun County Maternity and Child Health Care Hospital of Dezhou, Dezhou, Shandong 253799, China; ^7^Zhengzhou Key Laboratory of Children's Infection and Immunity, Children's Hospital Affiliated to Zhengzhou University, Zhengzhou 450000, China

## Abstract

**Objective:**

To identify the biological function and metabolic pathway of differential metabolites in follicular fluid of senile patients with kidney qi deficiency undergoing in vitro fertilization-embryo transfer (IVF-ET) and observe the effect of kidney-invigorating herbs on IVF outcomes in senile patients.

**Methods:**

A total of 95 women undergoing IVF treatment were recruited and divided into three groups, including 34 cases in the treatment group (the senile patients with kidney qi deficiency after the intervention of Chinese medicine), 31 cases in the experiment group (the senile patients with kidney qi deficiency of no intervention of Chinese medicine), and 30 cases in the control group (young women with infertility due to male factor). The three groups of women were treated with long protocol ovarian hyperstimulation; the treatment group was given Qi-Zi-Yu-Si decoction on the day of HCG downregulation. Their IVF clinical outcomes were observed. The metabolites changes of kidney qi deficiency syndrome were analyzed in follicular fluid metabolomics using liquid chromatography-mass spectrometry (UPLC-MS/MS).

**Results:**

The syndrome score of kidney qi deficiency syndrome in the treatment group was significantly improved after treatment (*P* < 0.01). Compared with the experiment group, the available embryo rate and implantation rate were increased, and the difference was statistically significant (*P* < 0.05). Progesterone, indoleacrylic acid, 2-propenyl 1-(1-propenylsulfinyl) propyl disulfide, N-acetyltryptophan, decanoylcarnitine, 20a-dihydroprogesterone, testosterone acetate, eicosatrienoic acid, 1H-indole-3-carboxaldehyde, choline, phosphorylcholine, and tryptophan were downregulated in the treatment group. Through pathway analysis, glycerophospholipid metabolism and steroid hormone biosynthesis were regulated in senile patients with kidney qi deficiency after Qi-Zi-Yu-Si decoction intervention.

**Conclusion:**

Qi-Zi-Yu-Si decoction can effectively improve the IVF outcome and clinical symptoms of senile patients. Follicular fluid metabolites were significantly changed in senile infertile women with kidney qi deficiency, and the mechanism by which kidney-invigorating herbs improve IVF treatment outcomes may be related to glycerophospholipid metabolism and steroid hormone biosynthesis. This study was registered in the Chinese Clinical Trials Registry Platform (ChiCTR1800014422).

## 1. Introduction

It is reported that 8% to 12% of couples of childbearing ages worldwide will be affected by infertility [1]. With the opening of China's “two-child policy,” the proportion of senile infertile couples has gradually increased [2]. At present, assisted reproductive technologies have developed rapidly, but the pregnancy rate in in vitro fertilization-embryo transfer (IVF-ET) cycles is still hovering between 30% and 40% [3]. The quality of oocytes has an important impact on fertilization and early embryonic development and is also one of the key factors affecting the therapeutic outcome of human assisted reproductive technologies. For senile infertile women, the decline in the number and quality of oocytes due to increasing age is the main reason for the low IVF success rate. However, at present, the evaluation of oocyte quality is mostly based on subjective experience, which has many limitations. Therefore, how to improve pregnancy outcomes in senile infertile women is currently one of the challenges facing the reproductive community.

Traditional Chinese medicine (TCM) holds that “kidney stores essence and dominates reproduction”, and kidney essence can promote the growth and reproductive function of the human body [4, 5]. The “Seven-Seven Theory” in the Internal Classic explains the changes in life activities dominated by the kidney essence with age, and infertility is mostly related to kidney qi deficiency [6]. Moreover, Professor Wang and his colleagues believe that kidney essence deficiency is the underlying cause of infertility in the elderly [7]. In the process of assisted reproductive technology treatment, the use of kidney-invigorating herbs to improve female reproductive function has achieved significant outcomes, but the mechanism of their action needs to be further studied.

Follicular fluid acts as the microenvironment for oocyte growth and development and the site of information exchange between oocytes and somatic cells, and changes in its composition reflect changes in follicular dynamics [8, 9]. With the decline of reproductive capacity, the composition of follicular fluid has also changed significantly [10]. The function and metabolic status of the human body can be analyzed from a holistic perspective using metabolomics. Metabolomics mainly studies the changes in metabolites produced by the body under different conditions, which can visually reflect the current metabolic status of organisms or cells, and the changed metabolites may be biomarkers for the occurrence and development of a disease [11–13]. In recent years, metabolomics based on ultra-high-performance liquid chromatography tandem mass spectrometry (UHPLC-MS) technology have been widely used due to their great advantages compared with nuclear magnetic resonance, GC-MS, and other technologies [14]. The ability of UHPLC-MS technology to analyze multiple metabolites through databases is important for in vivo metabolomics studies of untargeted metabolites in complex matrices. UHPLC-MS technology was used in this experiment to better detect and analyze differential metabolites.

In the early stage, two projects of National Natural Science Foundation of China have used nontargeted follicular fluid metabolomics based on UHPLC-MS technology to preliminarily screen and explore the biomarkers of kidney qi deficiency syndrome in the elderly [15]. The study found that the components of follicular fluid in elder women were significantly different from that in younger women. Non-targeted follicular fluid metabolomics has a wide coverage, but it has the weakness of low sensitivity and poor reproducibility. Targeted metabolomics with the low coverage has a wide linear range, good reproducibility and high sensitivity [16]. Semi-targeted metabolomics combines the advantages of nontargeted metabolomics and targeted metabolomics, which has high sensitivity, good reproducibility, and high coverage. In our study, semi-targeted metabolomics was used to explore the action mechanism of Qizi Yusi Decoction, a traditional Chinese medicine formula for tonifying kidney, in senile IVF patients with kidney qi deficiency. It is expected to find an effective method for improving the fertility of senile women and IVF treatment outcomes.

## 2. Materials and Methods

### 2.1. Materials

#### 2.1.1. Reagent

HPLC-grade methanol, acetonitrile, water, ammonium acetate, and formic acid were all supplied by Fisher Scientific (Fair Lawn, NJ, USA). The internal standards of chloramphenicol and clenbuterol were from Sigma Aldrich (St. Louis, MO, USA). Qi-Zi-Yu-Si decoction was obtained from the Affiliated Hospital of Shandong University of Traditional Chinese Medicine (Jinan, China) and authenticated by Professor Zhen-Gao Sun (Shandong University of Traditional Chinese Medicine, Jinan, China).

#### 2.1.2. Preparation of Qi-Zi-Yu-Si Decoction

Rehmannia glutinosa 15 g, staghorn cream 15 g, Cistanche deserticola 12 g, Yujin 12 g, Eclipta alba 12 g, Lycium barbarum 9 g, Ligustrum lucidum 9 g, Mulberry 9 g, Raspberry 9 g, Cuscuta chinensis 9 g, Whole lotus 9 g, Rosa laevigata 9 g, and Radix Glycyrrhizae 6 g are Chinese herbal pieces provided by the Pharmacy of the Affiliated Hospital of Shandong University of Traditional Chinese Medicine. According to the standard decoction of traditional Chinese medicine, soak in tap water for 1–2 hours; the water volume of one decoction is not more than 2–3 cm of the medicinal surface, and the water volume of the second decoction is not more than 1–2 cm of the medicinal surface; all the drugs are decocted at the same time; first decoct the drugs with fire, and then decoct slowly with gentle fire for 40–60 minutes. Take one dose daily, decocted in water, 30 to 60 minutes before breakfast and dinner.

In this study, the follicular fluid on the day of oocyte collection in women undergoing in vitro fertilization-embryo transfer (IVF-ET) was used.

#### 2.1.3. Subjects

Subjects who underwent IVF-ET for infertility were selected from the Reproductive Center of the Affiliated Hospital of Shandong University of TCM from October 2017 to January 2018. They were divided into the treatment group (the 34 senile patients with kidney qi deficiency after the intervention of Qi-Zi-Yu-Si decoction) and the experiment group (the 31 senile patients with kidney qi deficiency of no intervention of Qi-Zi-Yu-Si decoction). In addition, 30 healthy women who underwent IVF-ET due to male factors were selected as the control group. The present study was approved by the Reproductive Ethics Committees of the Affiliated Hospital of Shandong University of TCM (identifier: SDUTCM2017-E-0911).

#### 2.1.4. Diagnostic Criteria for Infertility

Women living without contraception for at least 12 months who are not pregnant are infertile [17].

#### 2.1.5. TCM Syndrome Differentiation Standard

It mainly refers to the third edition of the National Higher Traditional Chinese Medicine Education Textbook “Gynecology of Traditional Chinese Medicine” [18] and “Reference Standard for Syndrome Differentiation of TCM Deficiency Syndrome” [19]. In order to maximize the accuracy of syndrome differentiation of selected cases and avoid the inclusion of cases with both clinical and clip, the selected cases were independently differentiated by two sub-senior experts for the selected subjects, and the two syndromes coincided with each other, and those who did not coincide were eliminated. The syndrome differentiation criteria are as follows: main syndrome: long marriage infertility, pale menstrual color, and lumbosacral pain; concurrent syndrome: dizziness, tinnitus, loss of libido, fatigue, weak knees, or heel pain; tongue pulse: pale tongue and white fur; weak pulse. The above three syndromes are necessary.

#### 2.1.6. Inclusion Criteria for Senile Kidney Qi Deficiency

The inclusion criteria for senile kidney qi deficiency were as follows: 1. meeting the diagnostic criteria of infertility and TCM syndrome differentiation criteria of kidney qi deficiency syndrome; 2. age between 35 and 49 years; 3. did not use any steroidal hormone drugs three months before the test; 4. body mass index range 18.5–25 kg/m^2^.

#### 2.1.7. Inclusion Criteria for the Control Group

The inclusion criteria for the control group were as follows: 1. healthy women aged 21–34 years; 2. IVF-ET due to male factors; 3. have not used any steroidal hormone drugs 3 months before the test; 4. body mass index range 18.5–25 kg/m^2^.

#### 2.1.8. Exclusion Criteria

The exclusion criteria were as follows: 1. combined with immune diseases, infectious diseases, severe heart disease, and chronic wasting disease; 2. endometriosis; 3. chromosome abnormalities; 4. ovarian syndrome; 5. history of ovarian surgery; 6. history of radiotherapy and chemotherapy; 7. hysteroscopy showing uterine cavity lesions.

### 2.2. Methods

#### 2.2.1. Study Protocol

We followed the methods of Xiao et al. 2020 [20]. All the subjects were treated with recombinant human follicle-stimulating hormone (Gonal-F, Merck Serono, 75 IU/vial) after triptorelin acetate for injection (Daphnemaline, Ipsen Pharma Biotech, 0.1 mg/vial). Transvaginal ultrasound and blood sampling were used to detect the growth of follicles. The dosage of Gn was adjusted according to the number of follicles and speed of follicular growth. When the diameter of at least two follicles was ≥18 mm, 8000–10000 IU of hCG (hCG, Livzon Group, 2000 IU/vial) was intramuscularly injected. About 34–36 hours after hCG injection, transvaginal puncture was performed under the guidance of pelvic ultrasound for oocyte retrieval. Fertilization was performed at a concentration of 105 normal sperms/ml after oocyte retrieval. Qi-Zi-Yu-Si decoction, a traditional Chinese medicine for tonifying kidney, was administered from the beginning of the day of treatment to the day of hCG. The duration of administration of traditional Chinese medicine was about 24–26 days.

#### 2.2.2. Follicular Fluid Collection and Preservation

The first tube of yellowish, bloodless, and transparent follicular fluid was collected from all subjects on the day of oocyte retrieval and centrifuged for 10 min under 3000 × g. The supernatant was loaded into an Eppendorf tube, labeled, and directly frozen in a −80°C freezer.

#### 2.2.3. Clinical Observation Indicators

The cycle outcome of IVF-ET (number of oocytes retrieved, MII oocyte rate, IVF 2PN fertilization rate, ICSI 2PN fertilization rate, 2PN cleavage rate, available embryo rate, excellent embryo rate, implantation rate, and clinical pregnancy rate) and the changes of kidney qi deficiency syndrome score before and after treatment were observed.

#### 2.2.4. Sample Preparation

After sample thawing, 100 *μ*L of follicular fluid was mixed with 300 *μ*L of methanol and 5 *μ*L of internal standard solution. The mixture was centrifuged at 14000 g for 30 minutes. The supper-layer was dried using a nitrogen blower and then was dissolved using 100 *μ*L of mobile phase for analysis.

#### 2.2.5. Chromatographic Conditions

The separation was performed on a SCIEX ExionLC AD chromatography system (SCIEX, CA, USA) with a Waters HILIC (100 mm ∗ 2.1 mm, 1.7 *μ*m) column (Waters, Milford, MA, USA) at 40°C. Analysis was completed with a gradient elution of 0.1% formic acid in acetonitrile (*A*) and 10 mM ammonium acetate in water (B) within 19.0 min. The gradient program was 0.1% B at 0.01 min; 20% B at 8.0 min; 60% B at 12.0–16.0 min; and 0.1% B at 16.1 min. The flow rate was set to 0.4 mL/min. The sample injection volume was set to 10.0 *μ*L. All the samples were kept at 4°C during the analysis.

#### 2.2.6. Mass Spectrometry Conditions

The MS system was performed using a SCIEX QTRAP4000 (SCIEX, CA, USA). The multireaction monitor (MRM) and enhanced product ion (EPI) data were acquired in positive/negative electrospray ionization mode. The MRM transitions were extracted from the follicular fluid MS/MS spectra, which were acquired from TripleTOF5600 (SCIEX, CA, USA). Source parameters were defined as follows: temperature, 550°C; ion spray voltage, 5500 V (positive)/ − 4500 V (negative); nebulizer gas (Gas 1), 55 psi; heater gas (Gas 2), 50 psi; curtain gas, 25 psi; declustering potential, 60 V (positive)/ − 100 V (negative). Any MRM survey scan peak exceeding 150 cps was selected for dependent scan. 5 candidate ions were allowed per cycle. The collision energy was set to 35 V (positive)/ − 35 V (negative) with a collision energy spread of 15 V. All operations and data acquisition were controlled by the Analyst 1.6 software (SCIEX, CA, USA).

#### 2.2.7. Semi-Targeted Metabolomics Analysis

The LC-MS data files were imported into OS-Q software (SCIEX, CA, USA). The chromatographic peaks were extracted, respectively. Pareto scaling and multivariate analyses of log transformation were applied to the data processing. PLS-DA was performed to give the contribution of the lipids by VIP score. All the lipids with significance threshold satisfying corrected *P* value cut-off 0.05 in one-way ANOVA and VIP score >1 were considered as potential biomarkers. They were performed on MetaboAnalyst software 4.0 (Xia Lab at McGill University, Montreal, QC, Canada).

## 3. Results

### 3.1. Clinical Background

There was no significant difference in age, body mass index (BMI), duration of infertility, basal follicle-stimulating hormone (bFSH), basal luteinizing hormone (bLH), basal estradiol (bE2), gravidity, parity, and abortion rate between the treatment and control groups (*P* > 0.05) (Table 1).

### 3.2. Comparison of IVF Outcomes

The available embryo rate in the treatment group was higher than that in the experiment group, and the difference was statistically significant (*P* < 0.05); the MII egg rate, ICSI 2PN fertilization rate, and available embryo rate in the experiment group were lower than those in the control group, and the difference was statistically significant (*P* < 0.05); there were no significant differences among the three groups in IVF 2PN fertilization rate and 2PN cleavage rate (*P* > 0.05). The embryo implantation rate in the treatment group was significantly higher than that in the experiment group, and the difference had statistical significance (*P* < 0.05); the embryo implantation rate in the control group was higher than that in the experiment group, but there was no statistical significance between the control group and the treatment group (*P* > 0.05), and there was statistical significance between the control group and the experiment group (*P* < 0.05); the clinical pregnancy rate in the treatment group was higher than that in the experiment group, and the differences had statistical significance (*P* < 0.05); the number of oocytes retrieved and clinical pregnancy in the control group were higher than those in the experiment group, and the differences had statistical significance (*P* < 0.05) (see Table 2).

### 3.3. Comparison of Kidney Qi Deficiency Syndrome Score

In the treatment group, the TCM score on the HCG day after treatment was significantly lower than that on the regulation day, and the difference was statistically significant (*P* < 0.001) (see Table 3).

### 3.4. Multivariate Statistical Analysis

A large-scale multireaction monitor (MRM) was applied in the LC-MS detection. Typical chromatograms of follicular fluid are shown in Figure 1. Chromatographic peaks were then carried out for alignment and normalization, followed by multivariate statistical analysis. Partial least-squares discriminant analysis (PLS-DA), a supervised multivariate analysis, was employed for metabolomics study. As shown in the PLS-DA score plots, follicular fluid samples from the control group, the experiment group, and the treatment group were well separated into three categories (Figure 2), suggesting that metabolic perturbation significantly occurred in elder patients. A heatmap based on the intensity levels of the metabolites among the three groups is used to clearly characterize the follicular fluid profile of senile patients with kidney qi deficiency (Figure 3). All differentiated metabolites satisfying corrected *P* value cut-off 0.05 in one-way ANOVA were listed. The results showed that the contents of progesterone, indoleacrylic acid, 2-propenyl 1-(1-propenylsulfinyl) propyl disulfide, N-acetyltryptophan, decanoylcarnitine, 20a-dihydroprogesterone, testosterone acetate, eicosenoic acid, 1H-indole-3-carboxaldehyde, choline, phosphorylcholine, and tryptophan in the treatment group were downregulated after Qi-Zi-Yu-Si decoction intervention. Their MS/MS spectrum was compared with the reference MS/MS spectrum to eliminate the complex matrix interference of follicular fluid and confirm them. For example, the comparison spectrum of choline is shown in Figure 4. Through pathway analysis, after intervention with traditional Chinese medicine, glycerophospholipid metabolism and steroid hormone synthesis in patients were regulated, as seen in Figure 5.

## 4. Discussion

Since the age of 35, ovarian function and fertility of women gradually decline, and there are usually manifestations of infertility for several years before menopause [21]. The implantation rate and pregnancy rate of elderly women gradually decreased, but the spontaneous abortion rate gradually increased, of which the decrease in the number and quality of oocytes is considered to be the main reason [22].

In this study, we analyzed the differences in follicular fluid metabolites after the Qi-Zi-Yu-Si decoction intervention of IVF in senile patients with kidney-qi deficiency, explored and validated biomarkers of advanced age, and explored the semi-targeted metabolomics mechanism of fertility decline in elderly women. Combined with clinical data and metabolomics analysis, the available embryo rate and implantation rate in the treatment group were significantly improved (*P* < 0.05) (Table 2), and the symptoms of kidney qi deficiency were significantly improved (*P* < 0.01) (Table 3). The symptoms of “lumbosacral pain, dizziness, tinnitus, fatigue, loss of libido, weakness of the knee, or heel pain” manifested by kidney qi deficiency syndrome in patients after taking TCM Qi-Zi-Yu-Si decoction were significantly improved compared with those before treatment. The IVF outcome indicators tended to be close to those in the control group. As seen in Figure 2, the treatment group was close to the control group and showed a tendency of separation from the experiment group, indicating that the traditional Chinese medicine intervention had a certain effect by regulating the metabolites. It was found that the contents of metabolites were upregulated in the experiment group, compared with the control group, and downregulated close to that of the control group after the intervention of Qi-Zi-Yu-Si decoction in the treatment group. After pathway analysis, the differential metabolites were involved in glycerophospholipid metabolism and steroid hormone synthesis. These metabolites may be biomarkers of kidney qi deficiency syndrome in the elderly.

Traditional Chinese medicine has played an important role in the treatment of infertility in senile women, and tonifying the kidney and filling the essence have become the fundamental treatment to improve ovarian dysfunction. Many literature studies have confirmed that some active components in kidney-invigorating herbs have antiaging effects [23], mainly by regulating the function of the hypothalamic-pituitary-ovarian axis and overall adjusting reproductive endocrine levels, thereby improving the function of the ovary. Gao et al. used Bushen to significantly improve the symptoms of kidney deficiency in elderly female infertile patients after 3 months of treatment, and E2 and anti-Müllerian in vitro hormone levels were significantly improved compared with those before treatment [24]. Zuo and her colleagues evaluated the therapeutic effect of tonifying the kidney and regulating the week on poor ovarian response. The results showed that the number of oocytes retrieved, the number of MII eggs, the excellent embryo rate, and the clinical pregnancy rate of IVF cycles were significantly increased [25]. The above findings have consistently shown that kidney-invigorating herbs can improve female fertility, and Qi-Zi-Yu-Si is following the method of tonifying the kidney to fill in the essence.

Lipid metabolism including glycerophospholipid metabolism is considered to be one of the main factors affecting the developmental capacity of oocytes and embryos. The follicular fluid microenvironment has its unique lipid profile, providing specific conditions for the growth and development of oocytes [26]. Lipids in oocytes are mainly stored in lipid droplets (LDs) in the form of triglycerides (TG), which provide energy for the development and maturation of oocytes [27]. The most abundant intracellular lipid stored in oocytes is triacylglycerol (TAG), which can generate energy through the *β*-oxidation reaction of mitochondria during oocyte maturation [28]. The lipid content in the oocyte can reflect the extent of *β*-oxidation in this cell to maintain its role during fertilization and embryo development, and it can be argued that the higher lipid content reflects a greater reliance on fatty acids as substrates for energy production [29]. Bertuccez et al. did a prospective study in an attempt to find changes in the lipid composition of follicular fluid components in old and young women in order to discover potential lipid biomarkers of oocyte aging. The results showed that phosphatidic acid (PA), phosphatidylinositol (PI), monogalactosyldiacylglycerol (MGDG), phosphatidic acid (PG), sphingomyelin (SM), diacylglycerol (DG), triacylglycerol (TG), phosphatidylcholine (PC), phosphatidylethanolamine (PE), phosphatidylinositol phosphate (PIP), digalactosyldiacylglycerol (DGDG), and phosphatidylserine (PS) were increased in elder patients [30]. In our study, we found that the lipid content of oocytes was significantly downregulated after the intervention of Qi-Zi-Yu-Si decoction.

Progesterone, mainly secreted by the corpus luteum and placenta, is an intermediate in gonadal steroid hormone synthesis, which acts directly on various tissues to regulate reproductive function. It is mainly involved in the menstrual cycle and pregnancy of women as a hormone essential for embryo implantation and pregnancy maintenance. The regulation of progesterone on the selection, growth, and ovulation of dominant follicles is a complex process. The activity of adenylyl cyclase was inhibited by progesterone, resulting in a decrease in the concentration of cAMP to trigger oocyte maturation [31]. Some studies had shown that the fertilization rate is high when the level of progesterone in follicles is high [32]. However, Ben-Rafael et al. suggested that oocytes with high level of progesterone are often associated with dysplastic multinucleated embryos [33]. Asimakopoulos et al. found that embryo quality was not associated with the level of progesterone levels [34]. In our study, the level of progesterone in the treatment group was downregulated after Qi-Zi-Yu-Si decoction intervention and close to that of the control group. The alternate of the level of progesterone was related to steroidogenic metabolism. Therefore, the optimal concentration of progesterone had a positive effect on oocyte development. Overexposure of progesterone could result in a rapid decline in oocyte quality. Vogel et al. found that the level of ATP was low in the culture medium of streptococci with progesterone and testosterone acetate [35]. Previous study found that developmental defects in oocytes may be caused by the low level of ATP [36, 37]. In our study, the levels of progesterone and testosterone acetate were downregulated in the treatment group. The results displayed that Qi-Zi-Yu-Si decoction may play a role in increasing oocyte ATP levels and regulating energy metabolism by reducing the level of progesterone and testosterone acetate. Eicosatrienoic acid is one of the essential PUFAs in the human body. It was involved in linoleic acid metabolism. PUFAs are essential raw materials for the synthesis of the lipid rich shell layer during oocyte maturation [38], which suggests that PUFAs have an important role in oocyte development and maturation. Wei-Wen Chen et al. displayed that PUFAs play a key role in regulating *C. elegans* reproductive capacity [39]. Lipid peroxidation would increase in mouse embryos during culture with PUFA, resulting in decreased embryonic development. The effect of PUFAs can be attenuated by adding antioxidants to the medium [40]. In our study, the level of eicosatrienoic acid was downregulated after Qi-Zi-Yu-Si decoction intervention, indicating that Qi-Zi-Yu-Si decoction may play a role as an antioxidant in treatment.

Choline and phosphorylcholine are mainly derived from phosphatidylcholine (PtdCho). Choline is an important methyl donor in the metabolism of the liposome. The limit of methyl donor during follicular culture could result in a significant decrease in the polar body oocyte rate [41]. Phosphorylcholine is a metabolite of choline in the glycerophospholipid metabolic pathway. Phosphatidylcholine-specific phospholipase C (PC-PLC) cleaves PtdCho on the glycerophosphate bond to produce PCho and the second messenger DAG. PC-PLC plays an important role in cell apoptosis and cell survival as well as in a variety of disease processes. Previous studies have found that follicular PCho levels are higher in patients with endometriosis than in healthy women [42]. Wallace et al. also found that the contents of choline and its metabolites glycerophosphorylcholine and PCho were decreased in the undivided follicles of fertilized eggs [43]. It has also been shown that a decrease in PCho levels can increase the level of ceramide. The high level of intracellular ceramide could induce cell differentiation and/or apoptosis and inhibit cell proliferation [44,45]. Pontoizeau et al. found that the level of PCho in *C. elegans* increased with age, which was identified as a potential biomarker of aging in *C. elegans* [46]. In our study, both choline and PCho levels in follicular fluid were downregulated after Qi-Zi-Yu-Si decoction intervention. Qi-Zi-Yu-Si decoction may have a negative role in cell differentiation and/or apoptosis.

Decanoylcarnitine exists in tissues and body fluids in free and esterified forms, which is mainly related to energy metabolism. Disturbed carnitine metabolism may impair the reproductive potential of in vitro fertilization. In previous study, carnitine profiles in serum and follicular fluid showed that the levels of total carnitine, free carnitine, and acylcarnitine in patients with >9 oocytes and/or >6 embryos were lower than those of IVF patients with <9 oocytes and/or <6 embryos [47]. The intermediate of follicular fluid lipid metabolism is diacylglycerol (DAG), which is produced by hydrolysis of phosphatidylinositol (4, 5)-bisphosphate and PKC. The activation of PKC can regulate apoptosis [48]. PUFAs in follicular fluid produce large amounts of ATP through *β*-oxidative metabolism. Some studies have confirmed that fatty acids have an important role in obtaining the energy supply for oocyte and early embryo developmental competence [49]. The accumulation of acylcarnitines is considered to be a marker of mitochondrial dysfunction and impaired metabolism of cellular PUFAs, affecting energy metabolism. Decanoylcarnitine can inhibit the transport of mitochondrial fatty acids by inhibiting carnitine-acylcarnitine translocase (CACT). The high level of free fatty acids will result in oocyte mitochondrial and spindle abnormalities [29]. In addition, the high level of free PUFAs in follicular fluid can also lead to intrafollicular lipotoxicity and impair oocyte quality, thereby reducing fertility in dairy cows [50]. Free PUFAs are metabolized by carnitine-mediated oxidation. In conclusion, decanoylcarnitine is harmful to oocyte quality and fertility by affecting mitochondrial dysfunction and energy metabolism. In our study, the content of decanoylcarnitine and indoleacrylic acid in the treatment group was downregulated close to that of the control group after the intervention of Qi-Zi-Yu-Si decoction. Qi-Zi-Yu-Si decoction may reduce the accumulation of decanoylcarnitine and adjust the function and energy metabolism of mitochondria by interfering the oxidative metabolism of PUFAs to a certain extent.

In addition, the contents of tryptophan, N-acetyltryptophan, and 1H-indole-3-carboxaldehyde and 2-propenyl 1-(1-propenylsulfinyl) propyl disulfide were downregulated in the treatment group. Tryptophan can be used as effective antioxidants in the body, scavenging reactive oxygen species, reactive nitrogen species, and enhancing the body's protection against free radicals. N-acetyltryptophan is a metabolite of tryptophan. In our study, the contents of tryptophan and N-acetyltryptophan in the treatment group were downregulated close to that of the control group after the intervention of Qi-Zi-Yu-Si decoction. No studies related to 1H-indole-3-carboxaldehyde and 2-propenyl 1-(1-propenylsulfinyl) propyl disulfide have been found, and its mechanism of action needs to be discovered.

In conclusion, semi-metabolomics provides a new idea and method for exploring the specific biomarkers of fertility decline in elderly women and finding the corresponding TCM treatment and exploring its mechanism of action. In our study, follicular fluid semi-metabolomics was used to explore the action mechanism of Qi-Zi-Yu-Si decoction to improve IVF outcomes in elderly patients. The sample size needs to be enlarged to verify our study. In addition, we will combine metabolomics with proteomics to fuse various metabolic pathways and regulatory pathways to jointly elucidate the overall status of biological systems and construct the expression regulatory network of the final metabolites in the further study.

## Figures and Tables

**Figure 1:** The typical chromatograms of follicular fluid samples.

**Figure 2:** The partial least-squares discriminant analysis recognition based on the follicular fluid metabolomic profiling.

**Figure 3:** The hierarchical clustering heatmap of the metabolites.

**Figure 4:** The comparison spectrum of choline between the experimental and reference MS/MS spectrum.

**Figure 5:** The metabolic pathways related to senile patients with kidney qi deficiency, as analyzed by MetaboAnalyst.

**Table 1:** The clinical data of subjects (*x* ± *s*).

	Patients	Healthy women
Age (years)	37.76 ± 2.27	38.94 ± 2.52
Body mass index (kg/m^2^)	22.80 ± 1.69	22.77 ± 1.32
Duration of infertility (years)	3.06 ± 2.34	2.90 ± 3.28
Basal FSH (IU/L)	7.16 ± 1.92	7.75 ± 2.70
Basal LH (IU/L)	4.91 ± 2.24	5.29 ± 2.30
Basal E2 (ng/ml)	47.29 ± 23.10	46.94 ± 17.04
Number of pregnancies	2.03 ± 1.83	2.10 ± 1.40
Parity	0.74 ± 0.57	0.87 ± 0.50
Flow	1.24 ± 1.50	1.16 ± 1.21

FSH: follicle-stimulating hormone; LH: luteinizing hormone; E2: estradiol. Baseline characteristics were comparable between the two groups (all *P* > 0.05).

**Table 2:** The IVF outcomes among the three groups (%).

	Treatment group	Experiment group	Control group
Number of oocytes retrieved	11.21 ± 5.92	9.87 ± 4.92	15.90 ± 7.51
MII ovum rate	88.89% (24/27)	83.16% (79/95)	94.64% (53/56)
IVF 2PN fertilization rate	60.73% (215/354)	56.92% (111/195)	61.23% (229/374)
ICSI 2PN fertilization rate	83.33% (20/24)	83.54% (66/79)	60.38% (32/53)
2PN cleavage rate	97.87% (230/235)	95.58% (173/181)	96.15% (275/286)
Available embryo rate	55.22% (127/230)	43.93% (76/173)^∗^	53.82% (148/275)
High embryo rate	13.48% (31/230)	12.72% (22/173)	18.91% (52/275)
Clinical pregnancy rate	44.12% (15/34)	22.58% (7/31)	86.68% (26/30)
Implantation rate	35.71% (20/56)	17.02% (8/47)^∗^	52.67% (31/60)

IVF: in vitro fertilization; ICSI: intracytoplasmic sperm injection. ^∗^The difference between the treatment group and the experiment group was statistically significant (*P* < 0.05). The differences between the control and treatment groups and between the control and experiment groups were all statistically significant (*P* < 0.05).

**Table 3:** Comparison of TCM syndromes scores before and after treatment in the TCM intervention group (*x* ± *s*).

	Deregulation day	hCG day	T	*P* value
Treatment group	16.79 ± 2.83	9.59 ± 1.99	22.262	<0.001

## Data Availability

The datasets generated during the present study are available from the corresponding author upon reasonable request.
